# Analysis of Medication Rule of Primary Epilepsy Based on *Xiaocheng Yan's* Clinical Experience Collection of Epilepsy

**DOI:** 10.1155/2022/9539944

**Published:** 2022-06-25

**Authors:** Yu Zhang, Lin Tong, Guangkun Chen, Jingpeng Deng, Lei Zhang, Hongtao Li, Pengfei Chang

**Affiliations:** ^1^Institute of Information on Traditional Chinese Medicine, China Academy of Chinese Medical Sciences, Beijing 100700, China; ^2^Institute of Chinese Materia Medica, China Academy of Chinese Medical Sciences, Beijing 100700, China

## Abstract

**Objective:**

To explore and analyze the medication rule of Professor *Xiaocheng Yan* in the treatment of primary epilepsy, hoping to provide reference for the clinical treatment of primary epilepsy.

**Methods:**

Mining and analysis of Professor *Xiaocheng Yan* sorted out the medical cases of primary epilepsy in *Xiaocheng Yan's* clinical experience collection of epilepsy, extracted the traditional Chinese medicine (TCM) prescription data in the medical cases, standardized the obtained TCM prescription data, and used the data mining function integrated by the ancient and modern medical case cloud platform V2.3.5 to carry out frequency statistics, cluster analysis, association analysis, and complex network analysis on the TCM data, and the common herbs used by Professor *Xiaocheng Yan* in the treatment of primary epilepsy, properties and classifications of commonly used herbs, pairs of commonly used herbs, and core prescriptions were obtained.

**Results:**

A total of 39 cases, 228 medical records, and 230 prescriptions data of TCM were included. A total of 96 Chinese medicinal herbs were involved, and the total frequency of medication was 3,828. High-frequency herbs include Rhizoma Gastrodiae (Tianma) (222 times), Ramulus Uncariae cum Uncis (Gouteng) (220 times), Rhizoma Acori Tatarinowii (Shichangpu) (216 times), Rhizoma Pinelliae Praeparatum (Fabanxia) (207 times), Bombyx Batryticatus (Jiangcan) (206 times), and Periostracum Cicadae (Chantui) (181 times). The main properties and flavors of commonly used Chinese medicinal herbs were sweet, bitter, and pungent, which were mainly attributed to the four meridians of liver, lung, heart, and spleen. Commonly used couplet herbs were {Periostracum Cicadae (Chantui)} ≥ {Bombyx Batryticatus (Jiangcan)}, {Rhizoma Acori Tatarinowii (Shichangpu)} ≥{ Bombyx Batryticatus (Jiangcan)}, {Radix Bupleuri (Chaihu)} ≥ {Radix Scutellariae (Huangqin)}, {Rhizoma Gastrodiae (Tianma)} ≥ {Ramulus Uncariae cum Uncis (Gouteng)}, {Rhizoma Acori Tatarinowii (Shichangpu)} ≥ {Periostracum Cicadae (Chantui)}, {Ramulus Uncariae cum Uncis (Gouteng)} ≥ {Bombyx Batryticatus (Jiangcan)}, {Bombyx Batryticatus (Jiangcan)} ≥ {Rhizoma Gastrodiae (Tianma)}, {Rhizoma Acori Tatarinowii (Shichangpu)} ≥ {Ramulus Uncariae cum Uncis (Gouteng)}, etc. The core prescription composition was based on the addition and subtraction of Tianma Gouteng decoction and Erchen decoction. The main pharmacological mechanisms of core prescriptions are mainly reflected in antioxidation, enhancing GABA efficacy, and regulating NMDA channel and sodium channel, neuroprotection, and so on.

**Conclusion:**

Professor *Xiaocheng Yan*'s medication for the treatment of primary epilepsy was based on the principle of relieving wind and spasm, drying dampness and resolving phlegm, giving consideration to both Qi and blood, and harmonizing liver, lung, heart, and spleen.

## 1. Introduction

Epilepsy is a chronic brain disease caused by a variety of causes, which is characterized by recurrent, paroxysmal, and transient central nervous system dysfunction caused by excessive discharge of brain neurons [1]. The data of domestic epidemic survey show that there are more than 9 million epileptic patients in China, and about 400,000 new epileptic patients are added every year [2, 3]. Primary epilepsy refers to unknown etiology, and the brain cannot be found to cause seizures of abnormal function or structural damage, which may be related to genetic factors, generally in a specific age stage of the disease [4]. At present, there is no ideal eradication method for the treatment of this disease at home and abroad. In the treatment of epilepsy, antiepileptic drugs are mainly used to control and reduce seizures, and try to dispel the etiology, in order to maintain the normal brain nerve function [5]. Repeated frequent seizures and the long-term use of a variety of antiepileptic drugs (AEDs) will not only bring physical damage to patients with epilepsy but also affect the living conditions of study, employment, marriage, and childbearing to varying degrees, and bring economic burden and mental pressure to patients, family members, and society.

A large number of clinical research practice and experience summary of famous TCM in China show definite advantages in the treatment of epilepsy, which can improve the curative effect of AEDs, reduce the dosage of AEDs, lighten the side effects and adverse reactions of drugs, and, meanwhile, improve the quality of life and social life function of patients significantly [6]. The TCM medical record is a clinical document that records the actual operation of diagnosis and treatment by doctors in the process of clinical practice under the guidance of the theory of TCM. It is the record of clinical diagnosis and treatment of TCM. It preserves a large number of first-hand data of disease diagnosis and treatment, which reflects the clinical experience and treatment characteristics of doctors, and is an important resource for the inheritance of TCM academic research and famous TCM experience and academic thought. The in-depth study of TCM medical records can not only explore and summarize the principle of the development of the disease, but also summarize the previous clinical experience and have an in-depth understanding of the formation and development of TCM academic schools [7]. This paper uses modern information technology to analyze the prescription information of TCM in *Xiaocheng Yan*'s medical cases of primary epilepsy, and excavates its medication rule, in order to provide reference for the clinical treatment of epilepsy.

## 2. Materials and Methods

### 2.1. Data Sources

Data sources were derived from the medical data of primary epilepsy collected in *Xiaocheng Yan's* clinical experience collection of epilepsy, which published by TCM Ancient Books Publishing House in 2017, and its cover is shown in Figure 1. The selected cases were diagnosed clearly, with objective examination basis (EEG or MRI), complete data records, and continuous treatment and observation for more than one year. There were 100 medical cases in the book, including 9 cases of benign epilepsy in children, 13 cases of epilepsy caused by febrile convulsion, 11 cases of epilepsy caused by craniocerebral trauma, 4 cases of absence epilepsy in children, 35 cases of idiopathic epilepsy, and 28 cases of secondary epilepsy [8].

### 2.2. Inclusion and Exclusion Criteria

#### 2.2.1. Inclusion Criteria

① The disease diagnosis belongs to hereditary generalized epilepsy (Note: *Xiaocheng Yan's* clinical experience collection of epilepsy was called “idiopathic epilepsy.” In addition, it also includes the medical records diagnosed as “childhood absence epilepsy” in this book, which was “hereditary generalized epilepsy” according to the epilepsy classification standard of ILAE Classification of the Epilepsies Position Paper of the ILAE Commission for Classification and Terminology [9]). ② The disease diagnosis belongs to self-limiting focal epilepsy (Note: *Xiaocheng Yan's* clinical experience collection of epilepsy was called “children's benign epilepsy”); ③ the curative effect was cured, improved, and effective (Note: the curative effect referred to here was clearly stated in the book. In addition, according to the Diagnostic and Curative Effect Standard of TCM Disease and Syndrome [10], it was cured in the near future: compared with the intermittent time of attack before treatment, it was longer than that of the author for more than one year; Improvement: the symptoms of the attack were less than before, and the interval was obviously prolonged).

#### 2.2.2. Exclusion Criteria

① Epilepsy caused by central nervous system infection; ② epilepsy caused by hypoxia; ③ epilepsy caused by craniocerebral trauma; ④ epilepsy caused by central nervous system malformation; ⑤ epilepsy caused by shock; ⑥ epilepsy caused by brain tumor; ⑦ eclampsia (epilepsy caused by pregnancy induced hypertension); ⑧ invalid medical records (Note: for epilepsy caused by the above causes, *Xiaocheng Yan's* clinical experience collection of epilepsy has indicated a clear diagnostic basis).

Select medical records according to the above inclusion and exclusion criteria, split diagnosis times, extract prescription data of TCM, and use the function in Microsoft Excel 2019 to check the consistency of the data, check the inconsistencies, input the original data according to the original data, and then import the split medical records and prescription data into the ancient and modern medical records cloud platform V2.3.5.

#### 2.2.3. Data Normalization

The aliases and abbreviations of drugs are unified as the names of TCM written in the textbook “Chinese pharmacy” [11] (hereinafter referred to as “Chinese pharmacy”) in the thirteenth five-year plan of higher education of TCM published in August 2016. For example, Yuanshen was unified as Xuanshen, and Shanzhi was unified as Fructus Gardeniae (Zhizi) and so on.

### 2.3. Data Analysis

This study mainly uses the ancient and modern medical record cloud platform V2.3.5 software to mine the prescription data of TCM in the medical case of primary epilepsy. First of all, we used the Apriori algorithm to analyze the association rules of the herbs. Additionally, hierarchical clustering was used to classify high-frequency herbs. Finally, complex network analysis was used to confirm the core herbs prescribed for primary epilepsy treatment.

#### 2.3.1. Frequency Analysis

It carries on the frequency statistics to the herb, the meridian tropism, the medicinal property, and so on.

#### 2.3.2. Apriori Algorithm

The Apriori algorithm is a frequent itemset algorithm for mining association rules. We used it to illustrate the specific rules of TCM in primary epilepsy treatment. In our data, each herb was treated as a variable. The association analysis algorithm (confidence ≥0.7, support ≥0.7, and promotion >0.99) was used to mine the commonly used medicine pairs in the treatment of epilepsy. The confidence is the probability of the occurrence of the associated postitem in the case of the occurrence of the associated antecedent; the degree of support is the percentage of the number of simultaneous occurrence of the associated antecedent and postassociated items to the total number of events, that is, the probability of the simultaneous occurrence of the antecedent and postassociated items. The degree of promotion is the ratio of confidence to the probability of the occurrence of the postcorrelation item. The higher the support and confidence, the stronger the relationship between the antecedent and the postcorrelation, and the promotion degree >1 indicates that the relationship between the former and the latter is effective and strong; otherwise, it is invalid.

#### 2.3.3. Hierarchical Clustering Algorithm

In the hierarchical clustering algorithm, each herb was regarded as a cluster, and N clusters were combined to form a new class based on a similarity measure between objects. After testing, it is found that the absolute distance can get better classification effect than Euclidean distance and Chebyshev distance. The absolute distance was used to calculate the similarity between herbs. It can be described as calculating the polyline distance from one object to another, and sometimes, it can be further described as the average deviation of objects in each dimension of multidimensional space [12].

#### 2.3.4. Complex Network Analysis

The complex network analysis method was used to find the core prescription composition of epilepsy treatment. Complex network analysis is used to analyze complex interaction laws in complex systems in the real world based on a network model of nodes and edges. The complexities of diseases and human life systems are gradually being recognized, such that medical research from a network perspective has become an important topic in current medical research. We regarded the constituent herbs for primary epilepsy treatment as nodes and connections between two herbs as edges. Thus, we could rationalize all medical record data into a network of medicine nodes and edges using ancient and modern medical record cloud platform V2.3.5 and the hierarchical network algorithm.

Hierarchical network is a display of the network after hierarchical division. The core network can be extracted from the sparse network. The algorithm needs to specify two parameters: layer number (which determines the number of network graphs generated from the center of the network to the periphery of the network) and degree coefficient (which determines the density of the generated graph, the smaller the value, the more nodes are left). The specific parameter settings are as follows: [layout: circle; layer number: 3; degree coefficient: 1] [13].

## 3. Results

According to the above-mentioned criteria, 39 medical cases of primary epilepsy were selected. After separation, 228 medical records (total number of medical cases) and a total of 230 prescriptions were obtained.

### 3.1. Statistics of Commonly Used Chinese Medicinal Herb

The prescription data of TCM included in the medical cases of primary epilepsy involved a total of 96 kinds of TCM, and the total frequency of herb use was 3,828. The top 30 commonly used Chinese medicinal herbs with frequency ≥30 are listed in Table 1 according to the frequency from high to low. Among them, Rhizoma Gastrodiae (Tianma) have the highest use frequency, up to 222 times, and the use frequency (frequency = frequency/total number of medical cases) was 96.52%.

### 3.2. Attribute Statistics of Chinese Medicinal Herb

#### 3.2.1. Four Qi

Most of the prescriptions for primary epilepsy were mainly composed of mild, warm, and cold Chinese medicinal herb. Among them, the frequency of mild herb use was the highest (1012 times). The details are shown in Figure 2.

#### 3.2.2. Five Flavors

Most of the prescriptions for primary epilepsy were sweet, bitter, and pungent. Among them, pungent herbs were used most frequently (1569 times), as shown in Figure 3.

#### 3.2.3. Meridian Tropism

The main prescriptions for primary epilepsy were liver meridian and lung meridian. Among them, the herb use frequency of liver meridian was the highest (2064 times), as shown in Figure 4.

#### 3.2.4. Efficacy

The main prescriptions of primary epilepsy were relieved wind and spasm, removed dampness, and phlegm. Among them, the frequency of the use of antispasmodic herbs was the highest (428 times), as shown in Figure 5.

### 3.3. Clustering of Commonly Used Herbs

Cluster analysis of Chinese medicinal herb commonly used in medical cases of primary epilepsy was carried out. The cluster analysis of 30 Chinese medicinal herbs with frequency ≥30 times was carried out by using absolute distance and the longest distance method, as shown in Figure 6. The results showed that the above herbs could be divided into three categories according to the absolute distance of 140. The first category was Concretio Silicea Bambusae (Tianzhuhuang), Poria cum Ligno Hospite (Fushen), Radix Polygalae (Yuanzhi), Radix Et Rhizoma Glycyrrhizae (Gancao), and Pericarpium Citri Reticulatae (Chenpi). The second category was Fructus Gardeniae (Zhizi), Radix Scutellariae (Huangqin), Radix Bupleuri (Chaihu), Periostracum Cicadae (Chantui), Rhizoma Pinelliae Praeparatum (Fabanxia), Bombyx Batryticatus (Jiangcan), Rhizoma Acori Tatarinowii (Shichangpu), Rhizoma Gastrodiae (Tianma), and Ramulus Uncariae cum Uncis (Gouteng). The third category was subdivided with the absolute value distance of 100 and could be divided into three groups (group a: Radix Curcumae (Yujin), Radix Angelicae Sinensis<Danggui>, Radix Paeoniae Alba (Baishao), Radix Paeoniae Rubra<Chishao>), group b: Cortex moutan<Mudanpi>, Radix Codonopsis<Dangshen>, Raw Fossil Fragments<Shenglonggu>, Raw Concha Ostreae<Shenguli>, group c: Arisaema cum Bile<Dannanxing>, Fructus Aurantii Immaturus<Zhishi>, Poria<Fuling>, Rhizoma Chuanxiong<Chuanxiong>, Flos Chrysanthemi<Juhua>, Hawksbill Carapace<Daimao>, Semen Platycladi<Baiziren>, and Semen Ziziphi Spinosae<Suanzaoren>.

### 3.4. Commonly Used Medicine Pair

The relationship between Chinese medicinal herb and Chinese medicinal herb in the prescription data of primary epilepsy was analyzed by the method of association rules, and arranged in descending order according to the degree of support, as shown in Table 2. The results showed that the effective and strongly related herbs used frequently in the treatment of primary epilepsy were {Periostracum Cicadae (Chantui)} ≥ {Bombyx Batryticatus (Jiangcan)}, {Rhizoma Acori Tatarinowii (Shichangpu)} ≥ {Bombyx Batryticatus (Jiangcan)}, {Radix Bupleuri (Chaihu)} ≥ {Radix Scutellariae (Huangqin)}, {Rhizoma Gastrodiae (Tianma)} ≥ {Ramulus Uncariae cum Uncis (Gouteng)}, {Rhizoma Acori Tatarinowii (Shichangpu)} ≥ {Periostracum Cicadae (Chantui)}, {Ramulus Uncariae cum Uncis (Gouteng)} ≥ {Bombyx Batryticatus (Jiangcan)}, {Bombyx Batryticatus (Jiangcan)} ≥ {Rhizoma Gastrodiae (Tianma)}, {Rhizoma Acori Tatarinowii (Shichangpu)} ≥ {Ramulus Uncariae cum Uncis (Gouteng)}, and so on.

### 3.5. Core Prescription Composition

The composition of the core prescription used in the treatment of primary epilepsy was obtained through complex network analysis, as shown in Figure 7. The results showed that the herb components were Rhizoma Gastrodiae (Tianma), Ramulus Uncariae cum Uncis (Gouteng), Fructus Gardeniae (Zhizi), Radix Scutellariae (Huangqin), Poria cum Ligno Hospite (Fushen), Rhizoma Acori Tatarinowii (Shichangpu), Radix Polygalae (Yuanzhi), Bombyx Batryticatus (Jiangcan), Periostracum Cicadae (Chantui), Rhizoma Pinelliae Praeparatum (Fabanxia), Pericarpium Citri Reticulatae (Chenpi), Radix Bupleuri (Chaihu), Radix Paeoniae Alba (Baishao), Concretio Silicea Bambusae (Tianzhuhuang), Radix Curcumae (Yujin), Cortex moutan(Mudanpi), Cortex moutan (Mudanpi) and Radix Et Rhizoma Glycyrrhizae (Gancao). From the composition of the prescription, the core prescription used in the treatment of primary epilepsy was Tianma Gouteng decoction and Erchen decoction.

### 3.6. Allopathic Drugs Used in Primary Epilepsy

Many patients take one or more antiepileptic drugs for a long time before using Chinese medicine herbs. Although antiepileptic drugs (AEDs) can control seizures, it also induces a variety of adverse reactions such as mental, psychological, behavioral, cognitive function, and fatigue [14]. In addition, the adverse reactions of AEDs may have a cumulative effect, and the risk of adverse reactions in patients with epilepsy caused by multidrug combination was significantly increased [15]. This paper summarizes the mechanism and common adverse reactions of antiepileptic Western drugs involved in Professor *Xiaocheng Yan*'s treatment of primary epilepsy. The types, specific drugs, mechanism of action, adverse reactions, and literature sources of antiepileptic drugs are listed in Table 3. A total of 6 drugs were included such as carbamazepine, oxcarbazepine, clonazepam, valproic acid, levetiracetam, and topiramate.

In general, when serious adverse reactions occur in patients with epilepsy or seizures were effectively controlled, drug reduction or withdrawal was helpful to improve the quality of life of patients with epilepsy. Among patients without serious adverse reactions, seizure-free period (SFP) was the main reference to determine the stopping time of AED. The empirical treatment of SFP has been gradually reduced recent 2∼3 years in clinic. The speed of drug withdrawal should be considered after determining the stopping time, which refers to how much the drug gradient reduces and how long it takes to stop using drug completely. Withdrawal of AED too quickly may lead to withdrawal, and the frequency and severity of withdrawal were higher than those before treatment [21]. Professor *Xiaocheng Yan* usually adopts the scheme of reducing the dosage of Western medicine slowly in the treatment of primary epilepsy.

### 3.7. Analysis of the Main Pharmacological Mechanisms of Core Prescriptions

Through the analysis of the main pharmacological mechanisms of the core prescriptions used by Professor *Xiaocheng Yan* in the treatment of primary epilepsy, it can be found that different traditional Chinese medicines can enhance the antiepileptic effects through anti-inflammation, antioxidation, enhancing GABA efficacy, regulating NMDA channels and sodium channels, and neuroprotection (Table 4).

## 4. Discussion

Through the analysis, we can know that the high-frequency Chinese medicinal herbs commonly used in the treatment of primary epilepsy were Ramulus Uncariae cum Uncis (Gouteng), Rhizoma Gastrodiae (Tianma), Rhizoma Acori Tatarinowii (Shichangpu), Bombyx Batryticatus (Jiangcan), Radix Paeoniae Alba (Baishao), and cicada, which can calm the liver, relieve shock, and calm the mind. They are effective, safe, and can be taken for a long time without significant side effects.

The main symptoms of epilepsy were convulsions, “all the wind was dizzy, all belong to the liver,” “all the violent rigidity, all belong to the wind,” so the treatment must start from the liver and the wind. The liver qi was smooth, and the accumulation of depression was avoided, the first thing of treating the liver was to soothe the liver and regulate qi; therefore, Radix Bupleuri (Chaihu), Radix Curcumae (Yujin), and Fructus Aurantii Immaturus were frequently used; in addition, the liver stores blood, if blood deficiency or blood stasis, the liver wind was easy to move and twitch, so the liver must nourish blood and activate blood, medicinal Radix Paeoniae Rubra, Radix Angelicae Sinensis, Rhizoma Chuanxiong, promoting blood circulation can calming liver wind; Rhizoma Pinelliae Praeparatum (Fabanxia), Pericarpium Citri Reticulatae, Poria, Dannanxing dryness, and phlegm; and Suanzaoren, Fushen, Radix Polygalae awakening and enlightening. Cortex moutan, Gardenia jasminoides, and Radix Scutellariae (Huangqin) Georgi clear away heat, relieve the fire caused by qi depression, and dispel phlegm and heat with expectorant herbs. The herb properties with the functions of calming the liver and relieving wind, clearing heat, promoting blood circulation, dryness, dampness, and resolving phlegm were mainly mild, warm, and cold. Epilepsy was difficult to be treated, which may easily suffer from chronic disease, qi depression, fire injury, bitter cold medicine clearing away heat, purging fire, and strengthening Yin. The herb of pungent and warm can help yang to activate qi, relieve qi depression, and help spleen transport at the same time.

Another major symptom of epilepsy was unconsciousness, which was located in the heart, “the heart dominates the mind,” and the spirits were disturbed, resulting in loss of consciousness (coma). Phlegm heat and blood stasis were the most common causes of disturbance of the spirits, so resolving phlegm and promoting blood circulation, awakening, and opening the mind were the main points in the treatment of epilepsy. The liver wood transverses the spleen soil, the spleen loses healthy movement, the biochemical source of qi and blood was deficient, and the heart loses nourishment; the qi was abnormal, which affects the main qi function of the lung, and the pungent herb mainly enters the lung meridian; the herbs used mainly belong to the four meridians of liver, lung, heart, and spleen, which shows that Professor *Xiaocheng Yan*'s medication for epilepsy takes into account the characteristics of the liver, lung, heart, and spleen.

After cluster analysis of herbs, it was found that the treatment of epilepsy can be divided into three categories: dryness and dampness, relieve wind and relieve spasm, calm the heart, and tranquilize the mind. The first kind of herb has the main effect of dryness, dampness and phlegm, calm the heart, and calm the mind; the second kind of herb has the main effect of calm the liver and relieve wind, relieve spasm, and convulsions; the third kind of herb can regulate qi and calm nerves, calm shock, and resolve phlegm. The combination of Chinese medicinal herb commonly used by Professor *Xiaocheng Yan* in the treatment of primary epilepsy was found through association rules, included Ramulus Uncariae cum Uncis (Gouteng), Rhizoma Gastrodiae (Tianma), Rhizoma Acori Tatarinowii (Shichangpu), Polygala, Bombyx Batryticatus (Jiangcan), slough of cicada, Radix Bupleuri (Chaihu), Radix Scutellariae (Huangqin), and Radix Paeoniae Alba (Baishao). Yuan et al. [52] used the frequency analysis method in the ancient and modern medical case cloud platform (v2.2.2) to conduct data mining on the syndrome differentiation and medication rules of modern Chinese medicine in the treatment of epilepsy. They concluded that Rhizoma Acori Tatarinowii(Shichangpu) ranked first in the high-frequency herbs, which was also Xiaocheng Yan's clinical high-frequency medication. Wang et al. [53] used Apriori algorithm to mine the medication rule of TCM in the database for the treatment of epilepsy and found that the medicine pair with the highest reliability and strong correlation was {Pericarpium Citri Reticulatae (Chenpi)} ≥ {Rhizoma Pinelliae Praeparatum (Fabanxia)}, which reflected the importance of drying dampness and resolving phlegm in the treatment of epilepsy by TCM. However, it only carried out data mining from the perspective of the literature, and the results have limitations. In comparison, the innovation of this study was that taking primary epilepsy as the research object, starting from the clinical effective cases, and using the absolute distance algorithm, we have achieved a better classification, and the results also confirm that it was in line with the clinical characteristics of Professor *Xiaocheng Yan*.

Zhang et al. [54] used the complex network algorithm to mine and analyze the diagnosis and treatment data of YingaoYu's treatment of epilepsy, found the relationship between medicine symptom and medicine treatment, and compared the dose range of core herbs used by adults and children, respectively. However, she did not analyze the pharmacological mechanism of the core prescription. In our study, the core prescriptions used in the treatment of primary epilepsy were obtained by complex network analysis, which were based on Tianma Gouteng decoction and Erchen decoction, including Uncinaria, Rhizoma Gastrodiae (Tianma), Bombyx Batryticatus (Jiangcan), Periostracum Cicadae (Chantui), Gardenia jasminoides, and Radix Scutellariae (Huangqin), which can suppressing hyperactive liver, calming endogenous wind, and relieving spasm; Radix Bupleuri (Chaihu), Rhizoma Pinelliae Praeparatum (Fabanxia), Pericarpium Citri Reticulatae, Tianzhu Huang, Yuanjin phlegm and qi; Rhizoma Acori Tatarinowii (Shichangpu), Radix Polygalae, and Poria can calming the heart and tranquilizing the mind. On this basis, we analyzed the main pharmacological mechanism of the core prescription furtherly, which were mainly reflected in anti-inflammatory, antioxidation, enhancing GABA efficacy, regulating NMDA channel and sodium channel, neuroprotection, and so on.

## 5. Conclusions

In this study, by collecting and sorting out Professor *Xiaocheng Yan*'s medical records in the treatment of primary epilepsy, standardizing the data of Chinese medicinal herb, and using the method of data mining to analyze the prescription data obtained, we obtained Professor *Xiaocheng Yan*'s commonly used herbs, herb attribute characteristics, compatibility rule, and core prescription composition in the treatment of primary epilepsy. It was found that Professor *Xiaocheng Yan*'s treatment of primary epilepsy was based on the principle of relieving wind and relieving spasm, dryness and dampness, and resolving phlegm. In addition, the mechanism and common adverse reactions of anti-epileptic Western herbs involved in Professor *Xiaocheng Yan*'s medical cases of treating primary epilepsy were summarized, and the main pharmacological mechanisms of core prescriptions were summarized and analyzed. It was hoped that this conclusion can provide a useful reference for the clinical treatment of primary epilepsy.

## Figures and Tables

**Figure 1:** The cover of *Xiaocheng Yan's* clinical experience collection of epilepsy.

**Figure 2:** Radar chart of four properties of TCM in medical cases of primary epilepsy.

**Figure 3:** Radar chart of five flavors of TCM in medical cases of primary epilepsy.

**Figure 4:** Radar chart of channel tropism of TCM in medical cases of primary epilepsy.

**Figure 5:** Bar chart of efficacy distribution of TCM in medical cases of primary epilepsy.

**Figure 6:** Cluster analysis of Chinese medicine in medical cases of primary epilepsy.

**Figure 7:** Complex network analysis of the core prescription of primary epilepsy. Note. The boundary value represents the frequency of co-occurrence of the two nodes.

**Table 1:** Related information of Chinese medicinal herb contained in medical records of primary epilepsy (frequency ≥30).

Genus	Family	Herb Chinese-Latin-English	Frequency	Percentage (%)	Average	Min	Max	Standard deviation
Gastrodia	Orchidaceae	[Tianma] Rhizoma Gastrodiae (tall gastrodia tuber)	222	96.52%	12.38	6	20	2.94
Uncaria	Rubiaceae	[Gouteng] Ramulus Uncariae cum Uncis (gambir plant)	220	95.65%	10.42	6	20	1.91
Acorus	Araceae	[Shichangpu] Rhizoma Acori Tatarinowii (grassleaf sweetflag Rhizome)	216	93.91%	20.9	5	30	9.25
Pinellia	Araceae	[Fabanxia] Rhizoma Pinelliae Praeparatum (prepared pinellia tuber)	207	90.00%	8.5	5	15	2.17
Bombyx	Bombycidae	[Jiangcan] Bombyx Batryticatus (Stiff Silkworm)	206	89.57%	9.8	6	15	1.08
Cicada	Cicadae	[Chantui] Periostracum Cicadae (Cicada Slough)	181	78.70%	5.59	3	6	1.04
Scutellaria	Labiatae	[Huangqin] Radix Scutellariae (Baical skullcap root)	172	74.78%	10.77	6	15	2.4
Bupleurum	Umbelliferae	[Chaihu] Radix Bupleuri (Chinese Thorowax root)	171	74.35%	11.44	6	15	2.77
Gardenia	Rubiaceae	[Zhizi] Fructus Gardeniae (cape jasmine fruit)	160	69.57%	10.44	6	15	1.84
Glycyrrhiza	leguminous	[Gancao] Radix Et Rhizoma Glycyrrhizae (Liquorice root)	151	65.65%	5.79	3	15	1.22
Citrus	Rutaceae	[Chenpi] Pericarpium Citri Reticulatae (Dried Tangerine peel)	127	55.22%	7.73	6	10	1.98
Phyllostachys	Gramineae	[Tianzhuhuang] Concretio Silicea Bambusae (Tabasheer)	114	49.57%	9.12	6	15	2.17
Poria	Polyporaceae	[Fushen] Poria cum Ligno Hospite (Poria with hostwood)	112	48.70%	11.57	6	15	2.39
Polygala	Polygalaceae	[Yuanzhi] Radix Polygalae (thinleaf milkwort root)	99	43.04%	11.02	6	20	3.22
Cynanchum	Asclepiadaceae	[Baishao] Radix Paeoniae Alba (white peony root)	92	40.00%	11.71	6	15	2.89
Curcuma	Zingiberaceae	[Yujin] Radix Curcumae (turmeric root tuber)	88	38.26%	9.69	6	15	1.92
Paeonia	Ranunculaceae	[Mudanpi] Cortex moutan (tree peony bark)	73	31.74%	11.82	6	15	2.7
Angelica	Umbelliferae	[Danggui] Radix Angelicae Sinensis (Chinese Angelica)	70	30.43%	9.8	6	15	2.68
Arisaema	Araceae	[Dannanxing] Arisaema cum Bile (bile Arisaema)	61	26.52%	8.38	5	10	2.03
Paeonia	Ranunculaceae	[Chishao] Radix Paeoniae Rubra (red peony root)	59	25.65%	11.69	6	15	2.94
—	—	[Shenglonggu] Raw Fossil Fragments (raw keel)	57	24.78%	27.11	10	30	5.99
Ostrea	Ostreae	[Shenguli] Raw Concha Ostreae (Raw Oyster Shell)	57	24.78%	27.11	10	30	5.99
Ligusticum	Umbelliferae	[Chuanxiong] Rhizoma Chuanxiong (Szechwan Lovage Rhizome)	52	22.61%	18.08	6	30	8.92
Platycladus	Cupressaceae	[Baiziren] Semen Platycladi (Chinese Arborvitae Kernel)	49	21.30%	13.78	10	30	5.76
Citrus	Rutaceae	[Zhishi] Fructus Aurantii Immaturus (immature orange fruit)	47	20.43%	7.96	6	10	2
Zizyphus	Rhamnaceae	[Suanzaoren] Semen Ziziphi Spinosae (spine date seed)	46	20.00%	14.02	10	30	5.58
Poria	Polyporaceae	[Fuling] Poria (Indian bread)	45	19.57%	11.36	6	20	2.62
Salvia	Labiatae	[Dangshen] Radix Codonopsis (Tangshen)	39	16.96%	12.56	10	30	4.22
Hawksbill	Carapace	[Daimao] Hawksbill Carapace (hawksbill turtle shell)	37	16.09%	2.84	1.5	3	0.47
Chrysanthemum	Compositae	[Juhua] Flos Chrysanthemi (Chrysanthemum Flower)	35	15.22%	10	6	15	2.27

^*∗*^ *Note*. “—” means no.

**Table 2:** Commonly used herbs in the prescription of primary epilepsy.

No.	Items (LHS ≥ RHS)	Support degree	Confidence degree	Lifting degree
1	{Ramulus Uncariae cum Uncis (Gouteng)} ≥ {Rhizoma Gastrodiae (Tianma)}	0.95	0.99	1.03
2	{Rhizoma Gastrodiae (Tianma)} ≥ {Ramulus Uncariae cum Uncis (Gouteng)}	0.95	0.98	1.02
3	{Rhizoma Acori Tatarinowii (Shichangpu)} ≥ {Rhizoma Gastrodiae (Tianma)}	0.92	0.98	1.02
4	{Rhizoma Gastrodiae (Tianma)} ≥ {Rhizoma Acori Tatarinowii (Shichangpu)}	0.92	0.95	1.01
5	{Rhizoma Acori Tatarinowii (Shichangpu)} ≥ {Ramulus Uncariae cum Uncis (Gouteng)}	0.91	0.97	1.01
6	{Ramulus Uncariae cum Uncis (Gouteng)} ≥ {Rhizoma Acori Tatarinowii (Shichangpu)}	0.91	0.95	1.01
7	{Bombyx Batryticatus (Jiangcan)} ≥ {Rhizoma Gastrodiae (Tianma)}	0.89	0.99	1.03
8	{Rhizoma Gastrodiae (Tianma)} ≥ {Bombyx Batryticatus (Jiangcan)}	0.89	0.92	1.03
9	{Ramulus Uncariae cum Uncis (Gouteng)} ≥ {Bombyx Batryticatus (Jiangcan)}	0.88	0.92	1.03
10	{Bombyx Batryticatus (Jiangcan)} ≥ {Ramulus Uncariae cum Uncis (Gouteng)}	0.88	0.99	1.04
11	{Rhizoma Acori Tatarinowii (Shichangpu)} ≥ {Bombyx Batryticatus (Jiangcan)}	0.87	0.93	1.04
12	{Rhizoma Pinelliae Praeparatum (Fabanxia)} ≥ {Rhizoma Gastrodiae (Tianma)}	0.87	0.97	1.0
13	{Bombyx Batryticatus (Jiangcan)} ≥ {Rhizoma Acori Tatarinowii (Shichangpu)}	0.87	0.97	1.03
14	{Rhizoma Gastrodiae (Tianma)} ≥ {Rhizoma Pinelliae Praeparatum (Fabanxia)}	0.87	0.9	1.0
15	{Rhizoma Pinelliae Praeparatum (Fabanxia)} ≥ {Ramulus Uncariae cum Uncis (Gouteng)}	0.86	0.95	0.99
16	{Ramulus Uncariae cum Uncis (Gouteng)} ≥ {Rhizoma Pinelliae Praeparatum (Fabanxia)}	0.86	0.9	1.0
17	{Rhizoma Acori Tatarinowii (Shichangpu)} ≥ {Rhizoma Pinelliae Praeparatum (Fabanxia)}	0.84	0.9	1.0
18	{Rhizoma Pinelliae Praeparatum (Fabanxia)} ≥ {Rhizoma Acori Tatarinowii (Shichangpu)}	0.84	0.94	1.0
19	{Rhizoma Pinelliae Praeparatum (Fabanxia)} ≥ {Bombyx Batryticatus (Jiangcan)}	0.81	0.9	1.0
20	{Bombyx Batryticatus (Jiangcan)} ≥ {Rhizoma Pinelliae Praeparatum (Fabanxia)}	0.81	0.91	1.01
21	{Ramulus Uncariae cum Uncis (Gouteng)} ≥ {Periostracum Cicadae (Chantui)}	0.79	0.82	1.04
22	{Bombyx Batryticatus (Jiangcan)} ≥ {Periostracum Cicadae (Chantui)}	0.79	0.88	1.12
23	{Periostracum Cicadae (Chantui)} ≥ {Ramulus Uncariae cum Uncis (Gouteng)}	0.79	1.0	1.05
24	{Periostracum Cicadae (Chantui)} ≥ {Bombyx Batryticatus (Jiangcan)}	0.79	1.0	1.12
25	{Rhizoma Gastrodiae (Tianma)} ≥ {Periostracum Cicadae (Chantui)}	0.78	0.81	1.03
26	{Periostracum Cicadae (Chantui)} ≥ {Rhizoma Gastrodiae (Tianma)}	0.78	0.99	1.03
27	{Rhizoma Acori Tatarinowii (Shichangpu)} ≥ {Periostracum Cicadae (Chantui)}	0.77	0.81	1.03
28	{Periostracum Cicadae (Chantui)} ≥ {Rhizoma Acori Tatarinowii (Shichangpu)}	0.77	0.97	1.03
29	{Ramulus Uncariae cum Uncis (Gouteng)} ≥ {Radix Scutellariae (Huangqin)}	0.73	0.76	1.02
30	{Radix Scutellariae (Huangqin)} ≥ {Rhizoma Gastrodiae (Tianma)}	0.73	0.97	1.0
31	{Radix Scutellariae (Huangqin)} ≥ {Ramulus Uncariae cum Uncis (Gouteng)}	0.73	0.97	1.01
32	{Rhizoma Gastrodiae (Tianma)} ≥ {Radix Scutellariae (Huangqin)}	0.73	0.75	1.0
33	{Rhizoma Pinelliae Praeparatum (Fabanxia)} ≥ {Periostracum Cicadae (Chantui)}	0.72	0.8	1.02
34	{Ramulus Uncariae cum Uncis (Gouteng)} ≥ {Radix Bupleuri (Chaihu)}	0.72	0.75	1.01
35	{Radix Bupleuri (Chaihu)} ≥ {Rhizoma Gastrodiae (Tianma)}	0.72	0.97	1.0
36	{Radix Bupleuri (Chaihu)} ≥ {Ramulus Uncariae cum Uncis (Gouteng)}	0.72	0.97	1.01
37	{Rhizoma Gastrodiae (Tianma)} ≥ {Radix Bupleuri (Chaihu)}	0.72	0.75	1.01
38	{Periostracum Cicadae (Chantui)} ≥ {Rhizoma Pinelliae Praeparatum (Fabanxia)}	0.72	0.92	1.02
39	{Radix Bupleuri (Chaihu)} ≥ {Radix Scutellariae (Huangqin)}	0.7	0.95	1.27
40	{Radix Scutellariae (Huangqin)} ≥ {Radix Bupleuri (Chaihu)}	0.7	0.94	1.26

Note. Confidence ≥ 0.7, support ≥ 0.7, improvement ≥ 0.99.

**Table 3:** Mechanism of action of antiepileptic allopathic drugs.

No.	Category	Drugs	Mechanism of action	Side effects	References
1	Iminostilbene	Carbamazepine and oxcarbazepine	Inhibition of neuronal Na + currents	Bone marrow suppression, skin rash, and visual disturbances	(Ambrósio et al.) [16]
2	Benzodiazepine	Clonazepam	Agonist action at the GABAA receptor	Drowsiness, cognitive impairment, and euphoria	(Campo-Soria et al.) [17]
3	Aliphatic carboxylic acid	Valproic acid	Increases the synthesis of GABA	Blurred vision, hair loss, change in appetite, and constipation	(Rosenberg) [18]
4		Levetiracetam	It modulates synaptic neurotransmitter release through binding to the synaptic vesicle protein SV2A in the brain	Vomiting, tiredness, throat irritation, headache, diarrhea, and cough	(Noachtar et al.) [19]
5		Topiramate	It inhibits the AMPA subtype glutamate receptor and blocks Na + channels. It also increases GABA activity at GABA receptors	Dizziness, somnolence, diarrhea, depression, and nystagmus	(Kenna et al.) [20]

**Table 4:** Related active ingredients, functions, and possible mechanisms of Chinese herbs.

Chinese herbs	Active ingredients	Functions	Possible mechanism
[Tianma] Rhizoma Gastrodiae	Vanillyl alcohol Gastrodin Parishin Gastrodia elata extract 4-Hydroxybenzyl alcohol 4-Hydroxybenzaldehyde and analogs	Antioxidation Anticonvulsion Anti-inﬂammation Neuroprotection	(1) Adjust AP-1 expression through the JNK signaling pathway [22] (2) Preclude NMDA excitotoxicity [23] (3) Equalize the activity of GABA and glutamate [24] (4) Modulate the MAPK-associated inﬂammatory responses [25, 26] (5) Restrain Na_v_1.6 sodium currents [25, 26]
[Gouteng] Ramulus Uncariae cum Uncis	Rhynchophylline	Anticonvulsion Antioxidation Neuroprotection	(1) Regulate the expressions of MIF and cyclophilin A [27] (2) Reduce the expression of JNKp of MAPK signal pathways [28] (3) Restrain Na_v_1.6 I_NaP_ and NMDA receptor currents [23] (4) Reduce GFAP, S100 B proteins, and RAGE [29, 30] (5) Attenuate mossy ﬁber sprouting and astrocyte proliferation [29, 30] (6) Prevent neuron death [29, 30] (7) Modulate TLR and neurotrophin signaling pathways [31] (8) Restrain the expression of IL-1 and BDNF genes [31]
[Shichangpu] Rhizoma Acori Tatarinowii	Volatile oil a-asarone *β*-asarone Eudesmin a-asarone	Anticonvulsion Anti-apoptosis Neuroprotection	(1) Protect GABA-immunoreactive neurons [32] (2) Modulate GABA_A_ receptors then enhance tonic GABAergic inhibition [33] (3) Increase GABA, and reduce glutamate [32] (4) Increase neurotrophic factors by triggering the PKA signaling pathway [34] (5) Regulate Caspase-3 and Bcl-2 [34]
[Jiangcan] Bombyx Batryticatus	Beauvericin Ammonium oxalate Protein-rich extracts Other ethanol extracts	Anticonvulsion Anti-apoptosis Antioxidation Neuroprotection	(1) Modulate the PI3K/Akt signaling pathways [35] (2) Reduce IL-1*β*, IL-4, and TNF-a, and increase 5-HT and GABA [36] (3) Reduce intracellular Ca2+ levels to prevent neuronal signaling [36]
[Fabanxia] Rhizoma Pinelliae Praeparatum	Pinellia total alkaloids	Anticonvulsion	(1) Modulate GABAergic system [37] (2) Upregulate GABA_A_ receptors [37]
[Chantui] Periostracum Cicadae	Amino acid Trace element (Al/P/Ca/Mg) [38]	Anticonvulsion	Not clear
[Chaihu] Radix Bupleuri	Saikosaponin A	Anticonvulsion Neuroprotection	(1) Suppress NMDA receptor current, I_Nap_ [39–41] (2) Inhibit mTOR signaling pathway [39–41] (3) Increase Kv4.2-mediated IA [39–41]
[Huangqin] Radix Scutellariae	Wogonin	Spasmolysis	Enhancing expression of GABAA receptors [42]
[Zhizi] Fructus Gardeniae	Geniposide	Antioxidation	Decreasing TNF-a, IL-1*β* levels, and plasma expression of vascular pseudohemophilia factor [43]
[Chenpi] Pericarpium Citri Reticulatae	Tangeretin Nobiletin	Antiepileptic Antioxidation Neuroprotection	Decreasing TNF, IL-17, NF-*κ*B, and MAPK levels [44]
[Gancao] Radix Et Rhizoma Glycyrrhizae	Carbenoxolone	Antiepileptic	Reduce cortical glial fibrillary acidic protein and connexin 43 expression [45]
[Tianzhuhuang] Concretio Silicea Bambusae	Amino acid	Antiepileptic Anticonvulsion Neuroprotection	Reduce IL-1*β*, ICAM-1, IL-8, NF-*κ*B, GFAP, and TNF-a [46]
[Fushen] Poria cum Ligno Hospite	Triterpene	Tranquilization	Not clear
[Yuanzhi] Radix Polygalae	(3-sinapoyl) fructofu-ranosyl-(6-sinapoyl) glucopyranoside 3,4,5-trimethoxy-cinnamic acid (TMCA)	Neuroprotection Antiepileptic	(1) Reduce Bax and increase Bcl-2 [47] (2) Enhancing expression of GABAA receptors [48]
[Baishao] Radix Paeoniae Alba	Paeoniﬂorin	Anticonvulsion Neuroprotection	(1) Suppress the elevation of c-Fos protein and increase transthyretin and phosphoglycerate mutase 1 [49] (2) Suppress the elevation of glutamate-induced intracellular Ca2＋ [50]
[Yujin] Radix Curcumae	Curcumin	Antidepressant Improving- memory	Increase the expression of VEGF and its receptor FLK-1 [51]

## Data Availability

The data used to support the findings of this study are included within the article.
